# Artificial Intelligence Algorithm in Classification and Recognition of Primary Hepatic Carcinoma Images under Magnetic Resonance Imaging

**DOI:** 10.1155/2022/8950600

**Published:** 2022-06-07

**Authors:** Zehua He, Qingqiang Huang, Yingyang Liao, Xiaojie Xu, Qiulin Wu, Yuanle Nong, Ningfu Peng, Wanrong He

**Affiliations:** ^1^Department of General Surgery, Langdong Hospital of Guangxi Medical University, Nanning 530022, Guangxi, China; ^2^Department of Radiology, Guigang City People's Hospital, Guigang 537100, Guangxi, China; ^3^Department of Nutrition, Affiliated Tumor Hospital of Guangxi Medical University, Nanning 530021, Guangxi, China; ^4^Department of Hepatobiliary Surgery, Affiliated Tumor Hospital of Guangxi Medical University, Nanning 530021, Guangxi, China; ^5^Department of Gastroenterology, People's Hospital of Guangxi Zhuang Autonomous Region, Nanning 530021, Guangxi, China

## Abstract

This study aimed to discuss the application value of the bias field correction algorithm in magnetic resonance imaging (MRI) images of patients with primary hepatic carcinoma (PHC). In total, 52 patients with PHC were selected as the experimental group and divided into three subgroups: mild (15 cases), moderate (19 cases), and severe (18 cases) according to pathological grading. Another 52 patients with hepatic nodules in the same period were included in the control group. All the patients underwent dynamic contrast-enhanced (DCE) MRI examination, and the image qualities of MRI before and after bias field correction were compared. The DCE-MRI perfusion parameters were measured, including the transport constant Ktrans, reverse rate constant Kep, extravascular extracellular volume fraction (Ve), plasma volume (Vp), microvascular density (MVD), hepatic artery perfusion index (HPI), mean transit time of contrast agent (MTT), time to peak (TTP), blood volume (BV), hepatic arterial perfusion (HAP), full perfusion (FP), and portal venous perfusion (PVP). It was found that the sensitivity (93.63%), specificity (71.62%), positive predictive value (95.63%), negative predictive value (71.62%), and accuracy (90.01%) of MRI examination processed by the bias field correction algorithm were all significantly greater than those before processing (*P* < 0.05). The Ktrans, Kep, Ve, Vp, and MVD of patients in the experimental group were significantly larger than those of the control group, and severe group> moderate group> mild group (*P* < 0.05). HPI, MTT, TTP, BV, and HAP of patients in the experimental group were also significantly greater than those of the control group, which was shown as severe group > moderate group > mild group (*P* < 0.05). FP and PVP of the experimental group were significantly lower than those of the control group, and severe group < moderate group < mild group (*P* < 0.05). It was suggested that in MRI images of patients with PHC, the bias field correction algorithm could significantly improve the diagnosis rate. Each perfusion parameter was related to the pathological grading, which could be used to evaluate the prognosis of patients.

## 1. Introduction

Primary hepatic carcinoma (PHC) is one of the common malignant tumors in humans, and its mortality has been high [1]. According to the *Global Cancer Report 2014* issued by World Health Organization, the deaths due to liver cancer in China account for about 51% of that globally. It ranks second in the mortality of malignant tumors in rural areas in China and ranks the third in cities [2]. Hepatic carcinoma mostly occurs in the context of hepatitis and liver cirrhosis in China. Hepatitis, cirrhosis, and liver cancer are three steps experienced by many patients. Due to the poor reserve function of the liver, the antitumor immune function of the body is low, and the prognosis is also poor. Therefore, early diagnosis and effective treatment are the keys to improving the prognosis of patients with hepatic carcinoma [3, 4].

It has been shown that the histopathological grading of PHC is related to its degree of infiltration and distant metastasis and is the main influencing factor for its prognosis [5]. Thus, early diagnosis, accurate pathological grading, and timely treatment of PHC are the keys to prolonging the survival time of patients with liver cancer [6]. A hepatic biopsy is currently the gold standard for pathological grading of PHC. In addition to sampling errors, this invasive procedure may bring certain risks to patients, such as infection, hemorrhage, and even the spread of cancer cells. Therefore, it is particularly important to find a noninvasive, repeatable, and highly accurate examination method for clinical diagnosis and treatment. The most common diagnostic method for PHC is imaging examination. Currently, there are real-time ultrasound, histopathological examination, computed tomography (CT), magnetic resonance imaging (MRI), angiography, radionuclide imaging, and so on [7, 8].

Histopathological examination is the gold standard for the diagnosis of liver cancer, but it is necessary to combine it with clinical evidence in the pathological diagnosis. This is to comprehensively understand hepatitis B virus (HBV) and hepatitis C virus (HCV) infections in patients, the detection results of other tumor markers, and the imaging features of hepatic space occupying lesions [9]. With the rapid development of imaging technology, ultrasound and CT have become the common methods for clinical diagnosis, with easy operations and affordable cost. But if the imaging features of the hepatic space occupying lesions are not typical, it may be missed or misdiagnosed. MRI showed more and more prominent advantages in the diagnosis of PHC. Its good resolution of tissues, multisection, multiparameter observation, relatively nontoxic contrast agent, no radiation, nontrauma, and other characteristics make MRI the optimal choice for imaging diagnosis of PHC [10]. In the past, the diagnosis of PHC by MRI mainly focused on morphological changes according to the imaging features of the tumor, such as T2 weighted imaging (T2WI) hyperintensity, diffusion-weighted imaging (DWI) hyperintensity, pseudocapsule sign, and rapid wash-in and wash-out enhancement. Thereby, tumors can be easily distinguished from nontumor nodules, but the degree of pathological differentiation of tumors cannot be accurately inferred. With the continuous development of functional MRI technology, it can not only reflect histological characteristics such as microcirculation state and cell density of tumors but also reflect cell metabolism and biochemical information of tumors [11, 12]. This makes it possible to assess the pathological grading of PHC accurately using MRI.

Dynamic contrast-enhanced (DCE) imaging technology is a three-dimensional volumetric thin-slice scanning on the ground of the T1 weighted imaging (T1WI) sequence. The magnetic resonance contrast agent is injected into the venous bolus for repeated, multistage, and rapid scanning, which allows MRI to detect the situation of blood perfusion in internal organs and tissues and obtain multiple perfusion parameter information through relevant analysis by the processing software [13]. DCE-MRI can quantitatively evaluate the properties of blood vessels in tissues. It has been reported that this technique can accurately assess the level of tumor tissue microcirculation, as well as capillary permeability and hepatic artery blood supply ratio in hepatic malignant tumor tissues [14].

With the development and application of deep learning, deep learning models can replace traditional machine learning algorithms to automatically extract lesion features and achieve lesion classification and identification [15]. Hepatic MRI bias field correction is mainly to deal with image grayscale inhomogeneity caused by radiofrequency field inhomogeneity and other factors. The bias field correction algorithm utilized the estimation of the bias field and the corresponding spatial information, which could well deal with the impact of the image bias field on the segmentation. A hepatic bias field correction algorithm was put forward on the basis of grayscale preservation, which ensured that the corrected image retained the grayscale information of the original image to the greatest extent. Hepatic tissue segmentation was performed on the corrected images, and evaluation parameters like segmentation were used to reflect the performance of the bias field correction algorithm [16, 17]. To sum up, the hepatic MRI images of patients were processed under the bias field correction algorithm. The correlation was analyzed between multiphase DCE-MRI perfusion parameters and microvascular density (MVD) and pathological grading of PHC patients, which was to provide a certain theoretical basis for the diagnosis of PHC.

## 2. Materials and Methods

### 2.1. General Data of Patients

In this study, 52 patients with PHC admitted to the hospital from July 2019 to July 2021 were included in the experimental group. Another 52 patients with benign hepatic nodules admitted during the same period were chosen as the control group. The inclusion criteria of patients were as follows. The clinical symptoms and histopathological examination results of the patients were in line with the diagnostic criteria for PHC formulated in *PHC Diagnosis and Treatment Standards (Edition 2011)* [18]. The patients were willing to undergo a DCE-MRI examination, and they all had the first-time onset. All the patients and their families fully understood the situation and signed the informed consent, and this study was approved by the ethics committee of the hospital.

The exclusion criteria below were followed. Patients had cancer tissue infiltration or metastasis to other tissues or organs. Patients had dysfunction of other important organs, such as heart, lung, and kidney. Patients were complicated with severe immune system diseases, infectious diseases, or infectious diseases. Patients had contraindications to DCE-MRI.

The general data of the two groups of patients are shown in Table 1 for details. There was no significant difference in gender, age, and average age between the two groups (*P* > 0.05), which made the research was of comparability.

### 2.2. DCE-MRI Examination Method

The patients underwent a DCE-MRI examination after respiratory function training. Then 1.5 T MRI instrument was used, and the abdominal phased array coil was set to 8 channels. The abdominal belt was used to adjust the breathing state of the patients. Dynamic, fast, and enhanced scanning were performed, respectively. For scanning parameters, the field of view (FOV) was set to be (350 × 320) mm, time of echo (TE) was 1.5 ms, time of repetition (TR) was 4.2 ms, the interlayer spacing was 0, the layer thickness was 3.6 mm of the (320 × 195) matrix, and the number of excitations was 1. Only the flip angles (3°, 9°, and 25°) needed to be adjusted; during enhanced scanning, a total of 50 dynamic cycles were scanned, each cycle lasted about 6 seconds with 30 layers, and the whole process lasted about 5 minutes. The scanning parameters were set as follows: FOV = (215 × 284) mm, TE = 1.35 ms, TR = 3.2 ms, slice thickness = 3.24 mm, the matrix was sized as 521 × 521, and the number of excitation was 2. In the second scanning, the contrast agent gadolinium diamine of 0.2 mL/kg was injected from the median cubital vein at a rate of about 4 mL/s. In total, 20 mL of normal saline was injected at the same rate after the injection. DCE scanning required the patients to hold their breath throughout the procedure, with only light and rapid ventilation.

### 2.3. Bias Field Correction Algorithm

MRI bias field correction was an algorithm model under local coherence, global intensity, and spatial continuity information. It could keep the grayscale of images consistent before and after correction. Its objective function was shown as follows:

(1) $$\begin{array}{c} A_{\text{our}}=A_{\text{MPFCM}}+\gamma {\sum_{k=1}^{m}\left(1-h_{k}\right)}^{2}\\ =\sum_{i=1}^{d}\sum_{k=1}^{m}v_{ik}^{n}N_{ik}+\gamma {\sum_{k=1}^{m}\left(1-h_{k}\right)}^{2}. \end{array}$$

In the equation, *N*_*ik*_=∑_*a*∈*M*_*i*__*ω*_*kp*_[(*α*∑_*r*∈Ω_*T*_*i*_(*r*))‖*I*_*kp*_ − *h*_*r*_*u*_*i*_‖^2^+(1 − *α*)∑_*r*∈*O*_*k*__*K*(*r* − *k*)‖*I*_*kp*_ − *h*_*r*_*u*_*i*_‖^2^]. Ω represents the whole hepatic MRI image with background noise removed. *O*_k_ represents the local area of the grayscale value of the *k*-th pixel in the image. The membership template function was expressed as *V*=[*v*_*ik*_], which was used to describe the degree to which the pixel belonged to a certain cluster. *g*_*kp*_ ∈ [0,1] refers to the local spatial continuity weight, which stands for the influence of domain pixels. *T*_*i*_(*r*), *i*=1,2,…, *d*; *r*=1,2,…, *m* represents the label function, which was the intensity information for this image and guided the correct clustering. *I*_*kp*_ is the filtered image after background noises were removed, and it was obtained by multiplying the membership template with the original image. *U*={*u*_1_, *u*_2_,…, *u*_*d*_} is the clustering center. *α*(0 ≤ *α* ≤ 1) stands for a positive value to balance global intensity with local intensity. Parameter *n* > 1, *d* represents the number of clusters, and *m* is the total number of pixels in the image. The weighted function *K*(*r* − *k*) also represents a truncated Gaussian kernel function, which reflects the influence of the center pixel *r* on the surrounding pixels, and its value decreased as the distance from the center *r* to the neighbor pixels *k* increased. *γ* > 0 is to balance the effects of the intensity and intensity-preserving constraints mentioned above.

In the energy minimization equation, ∑_*r*∈Ω_*T*_*i*_(*r*)‖*I*_*kp*_ − *h*_*r*_*u*_*i*_‖^2^ refers to the global intensity of the image, which was to ensure the correct clustering of each pixel in the image. The term ∑_*r*∈*O*_*k*__*K*(*r* − *k*)‖*I*_*kp*_ − *h*_*r*_*u*_*i*_‖^2^ is used to guarantee the smoothness of the bias field under the local intensity of the image. ∑_*k*=1_^*m*^(1 − *h*_*k*_)^2^ is the constraint term proposed to ensure the grayscale of the image after bias field correction, ensuring the grayscale consistency of the image before and after bias field correction; that is, the corrected image (*I*/*h*) and the original image have the same grayscale. *g*_*kp*_ ∈ [0,1]*s* indicates the local spatial continuity weight, which was the influence of neighbor pixels. In the image space domain, a pixel *k* had a spatial coordinate (*n*_*k*_, *m*_*k*_), and a pixel *p* in the neighborhood had a spatial coordinate (*n*_*p*_, *m*_*p*_), then the local spatial weight information could be expressed as follows:

(2) $$\begin{array}{c} \omega_{kp}=\left\{\frac{-\exp\;\delta_{kp}}{\sum_{p\in M_{k}}\left(-\exp\;\delta_{kp}\right)}\right\}\exp\left(-\max\left(\left|m_{p}-m_{k}\right|,\left|n_{p}-n_{k}\right|\right)\right). \end{array}$$

In this equation,

(3) $$\begin{array}{c} \delta_{kp}=\frac{\left\{{\left[\left(\sum_{p^{\prime }\in \left(M_{k}/s\right)}{\left(I_{p^{\prime }}-I_{p}\right)}^{2}/\left(m_{k}-1\right)\right)+{\left(I_{p}-I_{k}\right)}^{2}\right]}^{\left(1/2\right)}-\left({\sum_{p\in M_{k}}\left[\left(\sum_{p^{\prime }\in \left(M_{k}/s\right)}{\left(I_{p^{\prime }}-I_{p}\right)}^{2}/\left(m_{k}-1\right)\right)+{\left(I_{p}-I_{k}\right)}^{2}\right]}^{\left(1/2\right)}/m_{k}\right)\right\}}{k}, \end{array}$$

where *k* represents a constant and *δ*_*kp*_ is the same when the image pixel value was multiplied by a constant.

The parameters *V*, *U*, and *h* could be obtained by minimizing the energy function *A*_our_. In this process, when solving one parameter, the other two parameters could be kept unchanged, which was the same as the standard D-means clustering method. Therefore, the parameters *V*, *U*, and *h* could be obtained by making the first derivative of the objective function *A*_our_ equal 0, respectively. The iteration of parameters was applied to estimate the bias field *h*, and the corrected image of the bias field could be obtained by *I*/*h*. Since the energy function *A*_our_ was a convex function to its variables, the method proposed here was robust to initialize parameters.

The membership function was solved at first.

The first-order partial derivative of the energy function *A*_our_ to the parameter *V* was computed, and the result was made equal to 0. Then the following equation was worked out:

(4) $$\begin{array}{c} \frac{\partial A_{\text{our}}}{\partial v_{ik}}=\sum_{i=1}^{d}\frac{\partial }{\partial v_{ik}}\sum_{k=1}^{m}v_{ik}^{n}N_{ik}=0. \end{array}$$

The variable *v*_*ik*_ was determined by the following equation:

(5) $$\begin{array}{c} {\left\{\frac{\partial v_{ik}}{\partial v_{ik}}=nv^{n-1}N_{ik}\right\}}_{v_{ik}=v_{ik}^{*}}=0. \end{array}$$

Because *V* in the energy function *A*_our_ needed to satisfy the constraint term ∑_*i*=1_^*d*^*v*_*ik*_=1, *v*_*ik*_ ∈ [0,1], the following equation was obtained:

(6) $$\begin{array}{c} v_{ik}^{*}={\left\{\sum_{a=1}^{d}\left[{\left(\frac{N_{ik}}{N_{ak}}\right)}^{1/n-1}\right]\right\}}^{-1}. \end{array}$$

Next, the clustering center was solved.

The first-order partial derivative of the energy function *A*_our_ to the parameter *U* was solved, and the result was made equal to 0, then the following equation was obtained:

(7) $$\begin{array}{c} \frac{\partial A_{\text{our}}}{\partial u_{i}}=\sum_{k=1}^{m}v_{ik}^{n}\frac{\partial N_{ik}}{\partial u_{i}}=0. \end{array}$$

The variable *u*_*i*_ was determined by the following equation:

(8) $$\begin{array}{c} {\left\{\frac{\partial A_{\text{our}}}{\partial u_{i}}=\sum_{k=1}^{m}v_{ik}^{n}\frac{\partial N_{ik}}{\partial u_{i}}\right\}}_{u_{i}=u_{i}^{*}}=0. \end{array}$$

Then the solution of *u*_*i*_ was calculated through the following equation:

(9) $$\begin{array}{c} u_{i}^{*}=\frac{\sum_{k=1}^{m}v_{ik}^{n}I_{k}\left(\left(1-\alpha \right)\left(h*K\right)+\alpha hT_{i}\right)}{\sum_{k=1}^{m}v_{ik}^{n}\left(\left(1-\alpha \right)\left(h^{2}*K\right)+\alpha h^{2}T_{i}\right)}. \end{array}$$

In the equation, the symbol ∗ refers to the convolution operator. *I*=∑_*p*∈*M*_*k*__(*ω*_*kp*_ · *I*_*kp*_)/∑_*p*∈*M*_*k*__*ω*_*kp*_, and *I* is the hepatic MRI image after background noises were removed. *I*_*k*_ represents the grayscale value of the *k*-th pixel in the filtered image *I*.

Finally, the bias field estimation was performed.

The energy function *A*_our_ was utilized to find the first-order partial derivative of the bias field parameter *h*, and it was set equal to 0, then equation equation could be worked out:

(10) $$\begin{array}{c} \frac{\partial A_{\text{our}}}{\partial h_{k}}=\sum_{i=1}^{d}\frac{\partial }{\partial h_{k}}\sum_{k=1}^{m}v_{ik}^{n}N_{ik}+\gamma \frac{\partial }{\partial h_{k}}\sum_{k=1}^{m}{\left(1-h_{k}\right)}^{2}=0. \end{array}$$

The variable *h*_*k*_ was determined by the following equation:

(11) $$\begin{array}{c} {\left\{\sum_{i=1}^{d}\frac{\partial }{\partial h_{k}}v_{ik}^{n}N_{ik}+\gamma \frac{\partial }{\partial h_{k}}{\left(1-h_{k}\right)}^{2}\right\}}_{h_{k}=h_{k}^{*}}=0. \end{array}$$

Therefore, the bias field *h*_*k*_ could be expressed as follows:

(12) $$\begin{array}{c} h_{k}^{*}=\frac{\alpha IA_{1}^{\left(1\right)}+\left(1-\alpha \right)\left(\left(IA_{2}^{\left(1\right)}*K\right)\right)+\gamma m}{\alpha A_{1}^{\left(1\right)}+\left(1-\alpha \right)\left(\left(IA_{2}^{\left(1\right)}*K\right)\right)+\gamma m}. \end{array}$$

In the equation (12), *A*_1_^(1)^=∑_*i*=1_^*d*^*v*_*i*_^*n*^*u*_*i*_*T*_*i*_, *A*_1_^(2)^=∑_*i*=1_^*d*^*v*_*i*_^*n*^*u*_*i*_^2^*T*_*i*_, *A*_2_^(1)^=∑_*i*=1_^*d*^*v*_*i*_^*n*^*u*_*i*_, *A*_2_^(2)^=∑_*i*=1_^*d*^*v*_*i*_^*n*^*u*_*i*_^2^, and *v*_*i*_ represents the membership degree of category *i*.

The experimental steps of this method are described in Figure 1.

1. Parameters *V*, *U*, and *h* and other parameters were initialized.
2. The membership template function *I*_mask_ was calculated.
3. The membership matrix was updated by multiplying equation (6) and the membership template function *I*_mask_.
4. The global variable *T*_*i*_(*r*) was updated.
5. The cluster center was updated via equation (9).
6. The bias field was updated through equation (12).
7. It was judged whether the convergence condition ‖*U*_new_ − *U*_old_‖ < *ε* was satisfied, where *ε* is a very small number. If it was satisfied, the calculation was stopped; if not, the calculation was continued with steps (3) to (6).

### 2.4. Pathological Judgment Standards

The patients in the experimental group were graded with Edmondson–Steiner's tumor pathological grading method [19]. The pathological grading was performed according to the size and morphology of tumor cells, nuclear size, basophilic cytoplasmic staining, nuclear staining depth, and cytoplasmic ratio. Differentiation grade I referred to the tumor cells arranged in fascicles; grade II referred to the tumor cells that were shown eosinophilic with rich cytoplasm, large nuclei, and dark staining. Grade III meant that the nuclear staining degree was deeper than that of grade II, and tumor giant cells appeared. For grade IV, the tumor cells were shown with less cytoplasm, larger nuclei, darker staining, lacking of intercellular connections, and low differentiation. According to the grading of pathological conditions, grade I belonged to the mild group, grades II-III were in the moderate group, and grade IV was in the severe group.

### 2.5. Observation Indicators

After the DCE-MRI scanning, processing software was used to analyze the measurement results as the two-chamber Tofts model was selected. During the period, necrotic tissue and blood vessel areas were avoided. The maximum microvascular density (MVD) was selected under a low power lens, while the number of microvessels was calculated under a high power lens. Double-blind counts were performed by two experienced radiologists, respectively; then the average value of MVD was taken. Three regions of interest were selected to measure the plasma volume (Vp), the extravascular extracellular volume fraction (Ve), and the transport constant Ktrans from intracellular to extracellular space. The reverse rate constant Kep from extracellular to intravascular space, hepatic artery perfusion index (HPI), mean transit time (MTT) of contrast agent, time to peak (TTP), blood volume (BV), full perfusion (FP), hepatic arterial perfusion (HAP), and portal venous perfusion (PVP) were used to determine the mean value of the three fields of view.

### 2.6. Statistical Methods

SPSS19.0 was applied for statistical analysis. The enumeration data were expressed as a percentage (%). The measurement data Ktrans, Kep, Ve, Vp, MVD, HPI, MTT, TTP, BV, FP, HAP, and PVP were expressed as mean ± standard deviation (*x*(_) ±*s*). The differences in the measurement data among the three groups were analyzed by variance analysis. The *t*-test and Pearson method were adopted to analyze the differences in measurement data between two groups. When *P* < 0.05, the difference was statistically significant.

## 3. Results

### 3.1. MRI Results of Liver Cancer Patients

Figure 2 shows the MRI images of a 64-year-old male patient with hepatic carcinoma. In Figure 2 below, the images a, b, c, and d were the MRI images of the PHC patient before being processed by the bias field correction algorithm, while images e, f, g, and h were the MRI images after the bias field correction algorithm processing. Images a and e were the MRI images, images b and f were the T1WI images, images c and g were the T2WI images, and images d and h were the DWI images.

After being processed by the bias field correction algorithm, the sensitivity, specificity, positive predictive value, negative predictive value, and accuracy of MRI examination were 93.63%, 71.62%, 95.63%, 71.62%, and 90.01%, respectively. These were all significantly greater than those before processing (*P* < 0.05), and the differences were of statistical significance, which could be discovered in Figure 3 for details.

### 3.2. Comparison of Ktrans, Kep, Ve, Vp, and MVD in Patients between the Two Groups

Ktrans, Kep, Ve, Vp, and MVD of patients in the experimental group were significantly greater than those in the control group (*P* < 0.05), suggesting that the differences were statistically significant. The details are shown in Figure 4.

### 3.3. Comparison of Ktrans, Kep, Ve, Vp, and MVD among Subgroups of Patients in the Experimental Group

With the pathological judgment standards, the patients in the experimental group were divided into three subgroups, namely, the mild group (15 cases), the moderate group (19 cases), and the severe group (18 cases). Ktrans, Kep, Ve, Vp, and MVD of the severe group > those of the moderate group > those of the mild group (*P* < 0.05), and all the differences were considered to be statistically significant.  Figure 5 shows the comparisons in detail.

### 3.4. Comparison of HPI, MTT, TTP, BV, FP, HAP, and PVP between the Two Groups of Patients

HPI, MTT, TTP, BV, FP, HAP, and PVP of patients were compared between the experimental group and the control group. HPI, MTT, TTP, BV, and HAP of patients in the experimental group were significantly higher than those of the control group (*P* < 0.05). FP and PVP of the experimental group were significantly lower than those of the control group (*P* < 0.05), which were all displayed in Figures 6 and 7.

### 3.5. Comparison of HPI, MTT, TTP, BV, FP, HAP, and PVP of Patients in Each Subgroup of the Experimental Group

The levels of HPI, MTT, TTP, BV, and HAP in the severe group > those in the moderate group > those in the mild group, *P* < 0.05. FP and PVP in the severe group < those in the moderate group < those in the mild group, *P* < 0.05. All the differences were of statistical significance, as observed in Figures 8 and 9.

### 3.6. Correlation Analysis of Hepatic DCE-MRI Perfusion Parameters and MVD in PHC Patients in Experimental Group

Hepatic DCE-MRI perfusion parameters Ktrans, Kep, Ve, Vp, HPI, MTT, TTP, BV, and HAP were positively correlated with MVD in the experimental group (*P* < 0.05). FP and PVP were negatively correlated with MVD in the group (*P* < 0.05). The differences were suggested to be statistically significant, as shown in Figure 10 in detail.

## 4. Discussion

DCE-MRI is a noninvasive imaging technique. It is to inject a paramagnetic contrast agent into the blood vessel after the T1 is shortened. If the imaging is repeated, the change in the signal intensity in the tissue can be measured. As the diffusion time of the contrast agent increases, the peripheral tissues are monitored. After being processed by professional software, the quantitative parameter technology can be applied to measure the pathological changes in blood perfusion, and this technology has been increasingly used to evaluate the vascular permeability and the tumor microcirculation [20, 21].

The level of MVD can reflect the formation of new blood vessels in tumor tissues. The permeability of new blood vessels in immature tumors is higher, and the permeability of new blood vessels is related to the dynamic enhanced detection method of DCE-MRI [22]. It has been reported that with the increase of the tumor tissue volume and the degree of differentiation of PHC, the arterial blood supply also increases accordingly, and the hepatic sinusoids may present a capillary state. Because the morphological basis of tumor tissue growth and infiltration lies in blood vessels, the new tumor tissues and blood vessels can provide nutrients. If the blood vessels are immature, their permeability is higher; the contrast agent injected in DCE-MRI examinations has a small molecular weight and is easy to exudate from blood vessels into the extracellular space [23, 24]. It was found in this research that the sensitivity, specificity, positive predictive value, negative predictive value, and accuracy of MRI diagnosis processed by the bias field correction algorithm were 93.63%, 71.62%, 95.63%, 71.62%, and 90.01%, respectively. All of the results were remarkably greater than those before processing as *P* < 0.05, which indicated that compared with the simple MRI images, the diagnostic performance of MRI under the bias field correction algorithm was more excellent.

The blood flow velocity, which can be reflected as Ktrans on the vascular permeability, is used to indicate the permeability of the microvessels in the cancer tissues. The rate of contrast agent infiltration from the extracellular space to the intravascular space of the blood vessels is regarded as Kep. The volume ratio of contrast agent leaks into the extravascular interstitial space to the extracellular volume is denoted as Ve. Ktrans, Kep, and Ve increase if the vascular permeability around the tumor tissue increases [25]. It was found that Ktrans, Kep, Ve, Vp, and MVD of the experimental group were significantly higher than those of the control group, *P* < 0.05 with statistically significant differences. In the subgroups, Ktrans, Kep, Ve, Vp, and MVD of the severe group > those of the moderate group > those of the mild group, and *P* < 0.05, indicating the differences were statistically significant. It was suggested that the quantitative perfusion parameters of PHC patients by DCE-MRI examination were greatly related to the MVD and lesion severity of patients, which was similar to the results of Liu and Qian [26].

Some scholars have reported that the hepatic lobular structure is damaged in patients with PHC, regenerative nodules and a large number of fibrous tissue hyperplasia are shown, and even the blood circulation path is changed [27]. The portal vein reflux is not smooth, the hepatic arteriovenous shunt occurs, the hepatic blood flow resistance increases, and the PVP can be reduced. Under the action of fibrous cords, hepatic veins and portal vein branches in patients with PHC are occluded and narrowed, and a large number of collagen fibers are deposited in the intercellular space of hepatocytes. The flow time of the contrast agent in the liver is prolonged, which increases MTT and TTP. As blood flow resistance increases, the blood flow through the portal vein decreases and the proportion of hepatic artery blood flow in the total hepatic circulation increases, resulting in a decrease in FP and an increase in HPI [28]. It was found that HPI, MTT, TTP, BV, and HAP of the experimental group were significantly higher than those of the control group (*P* < 0.05), while FP and PVP were significantly lower (*P* < 0.05); the differences were computed to be statistically significant. The levels of HPI, MTT, TTP, BV, and HAP in patients were shown that those of the severe group > the moderate group > the mild group (*P* < 0.05). In FP and PVP, those of the severe group < the moderate group < the mild group (*P* < 0.05); the differences were all of statistical significance. It could be suggested that the quantitative perfusion parameters of PHC patients by DCE-MRI were significantly related to the incidence of portal vein thrombosis in patients. With the aggravation of PHC lesions, the risk of portal vein thrombosis increased, HPI, MTT, TTP, BV, and HAP increased, while FP and PVP decreased. These results were exactly similar to the findings of Song et al. [29].

## 5. Conclusion

The hepatic MRI images of the patients were processed under the bias field correction algorithm. The correlation was also analyzed between the perfusion parameters of multiphase DCE-MRI and MVD and pathological grades of PHC patients to assist the clinical diagnosis of PHC. The results showed that the sensitivity, specificity, positive predictive value, negative predictive value, and accuracy of MRI were significantly improved after processing the bias field correction algorithm. DCE-MRI could evaluate the microcirculation status of PHC patients objectively and quantitatively, and the changes of quantitative perfusion parameters were significantly correlated with MVD and pathological grades. Quantitative perfusion parameters detected by DCE-MRI could evaluate MVD level and pathological grading, which was worthy of further promotion. However, only 52 cases with PHC were included in this work, the sample size was small and the source was single, which might affect the results. The image processing performance of the bias field correction algorithm also needed to be further analyzed. The research would need to be expanded in the future so as to verify the conclusion with more clinical experiments.

## Figures and Tables

**Figure 1:** Schematic diagram of the algorithm flow.

**Figure 2:** MRI images of a PHC patient before and after processing by the bias field correction algorithm.

**Figure 3:** MRI results before and after the bias field correction processing. A, B, C, D, and E indicated sensitivity, specificity, positive predictive value, negative predictive value, and accuracy, respectively. ^*∗*^Compared with those before processing, *P* < 0.05.

**Figure 4:** Comparison of Ktrans, Kep, Ve, Vp, and MVD between the two groups. ^*∗*^Compared with those of the control group, *P* < 0.05.

**Figure 5:** Comparison of Ktrans, Kep, Ve, Vp, and MVD in each subgroup of patients in the experimental group. ^*∗*^Compared with the data of the mild group, *P* < 0.05; ^#^compared with those of the moderate group, *P* < 0.05.

**Figure 6:** Comparison of HPI, MTT, TTP, and BV between the two groups of patients. ^*∗*^Compared with the responding data of the control group, *P* < 0.05.

**Figure 7:** Comparison of FP, HAP, and PVP between the two groups of patients. ^*∗*^Compared with the control group, *P* < 0.05.

**Figure 8:** Comparison of HPI, MTT, TTP, and BV of patients in each subgroup of the experimental group. ^*∗*^Compared with the data of the moderate group, *P* < 0.05; ^#^compared with the data of the moderate group, *P* < 0.05.

**Figure 9:** Comparison of FP, HAP, and PVP in each subgroup of the experimental group. ^*∗*^Compared with the data of the moderate group, *P* < 0.05; ^#^compared with the data of the moderate group, *P* < 0.05.

**Figure 10:** Correlation between hepatic DCE-MRI perfusion parameters and MVD in PHC patients in the experimental group. (a) showed the correlation between parameters Ktrans, Kep, Ve, and Vp and MVD, while (b) showed the correlation between parameters HPI, MTT, TTP, BV, FP, HAP, and PVP and MVD.

**Table 1:** General data of patients in the two groups.

Groups	Males	Females	Age	Average age
Experimental group	32 cases	20 cases	(19–76) years old	(57.14 ± 5.45) years old
Control group	30 cases	22 cases	(17–78) years old	(56.17 ± 5.29) years old
*P* value	0.081	0.094	—	0.083

## Data Availability

The data used to support the findings of this study are available from the corresponding author upon request.
